The article "miRNA-340 inhibits osteoclast differentiation via repression of MITF" was published in 2017. Journal: Biosci Rep.

# miRNA-340 inhibits osteoclast differentiation via repression of MITF

**DOI:** 10.1042/BSR20170302

**Published:** 2017-07-20

**Authors:** Hongying Zhao, Jun Zhang, Haiyu Shao, Jianwen Liu, Mengran Jin, Jinping Chen, Yazeng Huang

**Affiliations:** 1 Department of Pharmacy, Zhejiang Provincial People’s Hospital, Hangzhou, Zhejiang, China; 2 People’s Hospital of Hangzhou Medical College, Hangzhou, Zhejiang, China; 3 Department of Orthopedics, Zhejiang Provincial People’s Hospital, Hangzhou, Zhejiang, China

**Keywords:** miRNA-340, MITF, Osteoclast differentiation

## Abstract

Many miRNAs play critical roles in modulating various biological processes of osteoclast differentiation and function. Microphthalmia-associated transcription factor (MITF), a target of miR-340, served as pivotal transcription factor involved in osteoclast differentiation. However, the role of miR-340 and MITF during osteoclast differentiation has not yet been clearly established. Tartrate-resistant acid phosphatase (TRAP) staining assay was performed to identify osteoclasts differentiated from bone marrow-derived macrophages (BMMs). Quantitative reverse transcription PCR (qRT-PCR) or Western blotting was undertaken to examine the mRNA or protein expression respectively. Luciferase reporter assay was performed to investigate the interaction between miR-340 and MITF. MITF was knocked down and miR-340 was overexpressed and transfected into BMMs to detect their effects on osteoclast differentiation. Firstly, qRT-PCR analysis showed that miR-340 was down-regulated during osteoclast differentiation stimulated by macrophage-colony stimulating factor (M-CSF) and receptor activator of nuclear factor (NF)-κB (RANK) ligand (RANKL). Besides, we found that overexpression of miRNA-340 inhibited osteoclast differentiation and suppressed both the mRNA and protein level of MITF. Finally, Western blot and qRT-PCR analysis revealed that silencing MITF inhibited TRAP, calcitonin receptor, V-ATPase d2, and cathepsin K. miR-340 suppresses osteoclast differentiation by inhibiting MITF. Our findings may provide promising therapeutic targets for osteoclast-associated diseases.

## Introduction

Osteoclasts, responsible for bone resorption, are multinucleated cells (MNCs) differentiated from macrophage/monocyte precursors [1,2]. It is widely known that bone homeostasis is dependent on the balance between bone resorption mediated by osteoclasts and bone formation by osteoblasts [3]. Excessive bone resorption induced by overactivity of osteoclasts is often associated with bone loss-related diseases including osteoporosis, rheumatoid arthritis, periodontal disease, multiple myeloma, and metastatic cancers [4,5]. Thus, there is an urgent need for elucidating the molecular mechanism underlying osteoclast differentiation.

MicroRNAs (miRNAs), widely found in eukaryotes, are endogenous small non-coding RNAs of 19–25 nucleotides and highly conserved during biological evolution [6]. miRNAs can play important regulatory roles in cleavage and transcriptional repression [7]. Recent studies have reported that many miRNAs have been identified to involve in bone metabolism and osteoclast differentiation [8]. MiRNA-340 (miR-340), a specific miRNA, is implicated in diverse cancers including gastric [9], ovarian [10], breast [11], colorectal cancer [12], and others. Besides, Ma et al. [13] has presented evidence that miR-340 was down-regulated during osteoclast differentiation using microarray analysis, which was associated with the progression of osteoporosis. However, little literature concerning the precise role of miR-340 implicated in osteoclastogenesis has been published.

Goswami et al. [14] has presented that miR-340 could interact with the two binding sites on the 3′ untranslated region (UTR) of microphthalmia-associated transcription factor (MITF), thus leading to the degradation of MITF and a decline in the expression and transcriptional activity of MITF. Several lines of evidence has indicated that MITF served as pivotal transcription factor involved in osteoclast differentiation [5]. In addition, MITF was reported to play significant roles in the survival of osteoclast precursors [6] and implicate in the regulation of osteoclast differentiation markers including tartrate-resistant acid phosphatase (TRAP) [15], cathepsin K [16], chloride channel 7 (CLCN7), osteopetrosis-associated transmembrane protein 1 (Ostm1) [17], and osteoclast-associated receptor (OSCAR) [18].

In the current study, we hypothesized that miR-340 may regulate osteoclast differentiation by interacting with MITF. Our study provides the first evidence that overexpression of miR-340 interferes with the expression of MITF, resulting in an inhibition of osteoclast differentiation. These findings demonstrate not only the negative regulation of MITF by miR-340 but also the inhibitory effect exerted by miR-340 on osteoclast differentiation, which may provide possible therapeutic target for osteoclast-related diseases.

## Materials and methods

### Cell lines and culture

HEK293T cells were obtained from the American Type Culture Collection (ATCC, Manassas, U.S.A.). Cells were maintained in Dulbecco's modified Eagle's medium (DMEM, Gibco BRL, U.S.A.) supplemented with 10% fetal bovine serum (FBS, Gibco BRL, U.S.A.), penicillin (100 U/ml), and streptomycin (100 mg/ml) (Macgene Biotechnology Ltd., China) in humidified air with 5% CO_2_ at 37°C.

### Bone marrow-derived macrophages preparation and differentiation

C57BL/6 mice (6–8 weeks old) were obtained from Laboratory Animal Center of Shanghai Institutes for Biological Science. All animal experiments were performed in accordance with National Institutes of Health Guide for the Care and Use of Laboratory Animals. For preparation of bone marrow cells, mice were killed by cervical dislocation. After that, femurs and tibias were separated and both ends were cut off. Subsequently, the bone marrow was flushed out with cold PBS containing 2% FBS by a 25-gauge syringe. Then erythrocytes were lysed by M-lysis buffer (R&D Systems, U.S.A.).

To prepare osteoclast precursor cells bone marrow-derived macrophages (BMMs), bone marrow cells were maintained overnight in α-MEM consisting of 10% FBS in humidified air with 5% CO_2_ at 37°C. Then non-adherent cells were harvested in α-MEM supplemented with 10% CMG14-12 culture supernatant (source of macrophage-colony stimulating factor (M-CSF)) [19]. After 3 days of incubation, the adherent cells served as BMMs. For osteoclast differentiation *in vitro*, BMMs were maintained in 96-well plates (1.5 × 10^4^ cells/well) in α-MEM in the presence of M-CSF (50 ng/ml) and receptor activator of nuclear factor (NF)-κB (RANK) ligand (RANKL) (50 ng/ml) for 3 days.

### TRAP staining

Briefly, control BMMs or infected BMMs following treatment with or without M-CSF and RANKL were fixed with 4% paraformaldehyde and washed with PBS. Then BMMs were stained for TRAP activity by a leucocyte acid phosphatase kit (Sigma–Aldrich, U.S.A.) under the manufacturer’s protocol. TRAP-positive MNCs with more than three nuclei were counted as osteoclasts.

### Real-time quantitative reverse transcription PCR (qRT-PCR)

For mRNA expression, total RNA was isolated from BMMs using Trizol reagent (Invitrogen, U.S.A.) and then reverse transcribed into cDNAs using an ABI High Capacity cDNA RT Kit (Life Technologies, U.S.A.) according to the manufacturer’s instructions. qRT-PCR was performed to amplify the cDNA templates by SYBR Premix Ex TaqTM II Kit (TaKaRa). The specific primer sequences for miR-340, MITF, TRAP, calcitonin receptor, V-ATPase d2, and cathepsin K were introduced as previously published [13,19–21]. The relative mRNA expression levels were calculated by the 2^−ΔΔ^*C*^_t_^ method and normalized to GAPDH.

### Overexpression of miR-340 and retroviral gene transduction in BMMs

In brief, to overexpress miR-340 in BMMs, primary miR-340 sequence was synthesized, cloned into the pBABE retroviral vector, and packaged into retroviral vector by transfection into Phoenix A cells to generate pBABE-340 vector. BMMs were then incubated with the viral supernatants of pBABE or pBABE-340 in the presence of M-CSF (50 ng/ml) and polybrene (6 μg/ml) for 8 h. The expression of miR-340 in BMMs transfected with empty pBABE vector or pBABE-340 vector was examined by qRT-PCR and Western blot.

### 3′UTR luciferase reporter assay

MITF 3′UTR was amplified by PCR and then cloned into pGL3 vector. For luciferase assay, HEK293T cells (2 × 10^4^ cells per well) were seeded in 24-well plates and cultured for 24 h. After the cells reached 80% confluence, the cells were cotransfected with wild-type (wt) or mutant MITF 3′UTR luciferase reporter plasmids, together with control mimics or miR-340 mimics (GenePharma, China) by Lipofectamine 2000™ (Invitrogen, U.S.A.). After transfection, cells were subjected to luciferase assays by using the Dual-Luciferase Reporter Assay System (Promega, U.S.A.) following the manufacturer’s protocol. Firefly luciferase activity was normalized to *Renilla* luciferase activity.

### Western blot

Western blot was performed to detect the protein expression level of MITF. In brief, the proteins were isolated from BMMs transfected with empty pBABE vector, pBABE-340 vector, negative control siRNA (control) or MITF siRNA (si-MITF) in lysis buffer respectively. After that, equal proteins were separated by 10% SDS/PAGE gels and electroblotted onto PVDF membranes (Millipore, U.S.A.). After blocking the nonspecific binding sites with 5% fat-free milk, the membranes were incubated with primary antibody against MITF (Cell signaling, U.S.A.) overnight at 4°C, followed by further 1 h of incubation with secondary antibody horseradish peroxidase-conjugated goat anti-rabbit IgG. β-Actin served as the loading control. Blots were examined by an Enhanced Chemiluminescence (ECL) Detection kit (Pierce Biotechnology, U.S.A.) and the band intensity was analyzed by Image-Pro Plus 6.0 software.

### Small-interfering RNA (siRNA) transfection

si-MITF and scramble siRNA (control) were designed and synthesized by GenePharma (Shanghai, China). The siRNAs were transfected into BMMs by Lipofectamine 2000™ (Invitrogen, U.S.A.). qRT-PCR was performed to examine the knockdown efficiency.

### Statistical analysis

All data were analyzed by SPSS 16.0 (SPSS Inc, U.S.A.). Statistical differences between two groups were analyzed using Student’s *t*-test. The data are presented as the mean ± SD. All experiments were repeated at least three times. *P*<0.05 was regarded statistically significant.

## Results

### miR-340 was down-regulated during osteoclast differentiation induced by M-CSF and RANKL

M-CSF and receptor activator of RANKL are two critical cytokines involved in osteoclast differentiation. To investigate the effect of RANKL and M-CSF on osteoclast differentiation, BMMS were isolated from mice, and cultured in the absence or the presence of M-CSF (50 ng/ml) and RANKL (50 ng/ml) for 72 h. TRAP staining analysis revealed that BMMs stimulated with M-CSF and RANKL were differentiated into more TRAP-positive osteoclasts than that without treatment of M-CSF and RANKL (Figure 1A), indicating treatment with M-CSF, and RANKL may serve as osteoclastogenesis condition. To identify the miRNA expression profile of miR-340 during osteoclast differentiation, BMMs were cultured in the absence or the presence of M-CSF (50 ng/ml), and RANKL (50 ng/ml) for 0, 24, 48, and 72 h respectively. Statistical analysis of qRT-PCR demonsrated that relative expression level of miR-340 in BMMs treated with M-CSF and RANKL was down-regulated in a time-dependent manner. However, no obvious alteration of miR-340 expression was observed in BMMs without treatment of M-CSF and RANKL (Figure 1B). Our results indicated that upon stimulation of BMMs with M-CSF and RANKL, the relative expression level of miR-340 was down-regulated.

**Figure 1:** MiR-340 was down-regulated during osteoclast differentiation induced by M-CSF and RANKL (**A**) BMMS were isolated from mice and cultured in the absence or the presence of M-CSF (50 ng/ml) and RANKL (50 ng/ml) for 72 h. TRAP-positive (pink to purple) MNCs with more than three nuclei were counted as mature osteoclasts. (**B**) BMMs were cultured in the absence or the presence of M-CSF (50 ng/ml) and RANKL (50 ng/ml) for 0, 24, 48, and 72 h respectively. The relative expression of miR-340 was detected by qRT-PCR. *P<0.05 and **P<0.01 versus the group (without stimulation of M-CSF and RANKL).

### Overexpression of miRNA-340 inhibited osteoclast differentiation

In an effort to explore the potential role of miR-340 during osteoclast differentiation, a pBABE-340 retroviral vector, a pBABE vector carrying primary miR-340 sequence, was generated to overexpress miR-340. BMMs were transfected with the pBABE or pBABE-340 viral supernatants in the presence of 50 ng/ml M-CSF and 6 μg/ml polybrene for 8 h. Data of qRT-PCR assays showed that the relative expression of miR-340 was up-regulated significantly in BMMs transfected with pBABE-340 retroviral construct compared with that in pBABE-tranduced BMMs (Figure 2A). After the viral supernatants of pBABE or pBABE-340 were removed, BMMs were differentiated into osteoclasts in the presence of M-CSF and RANKL for 24 h. As shown in Figure 2(B), TRAP-positive MNCs that counted as osteoclasts decreased greatly in number, suggesting that the suppressive effect of miR-340 on osteoclast differentiation in BMMs. Furthermore, qRT-PCR was also performed to assess the relative expression levels of osteoclast marker genes TRAP, calcitonin receptor, V-ATPase d2, and cathepsin K. As expected, these osteoclast-specific genes were down-regulated in response to overexpression of miR-340 (Figure 2C). Based on these findings, our results revealed that overexpression of miRNA-340 inhibited osteoclast differentiation.

**Figure 2:** Overexpression of miR-340 inhibited osteoclast differentiation (**A**) The relative expression of miR-340 in BMMs transfected with pBABE or pBABE-340 retroviral construct was detected by qRT-PCR assays. (**B**) After the pBABE or pBABE-340 viral supernatants were removed, BMMs were cultured in osteoclastogenesis condition (M-CSF + RNAKL) for 24 h. Number of TRAP-positive osteoclasts in each well and representative images of TRAP positive (pink or purple) BMMs are shown. (**C**) The relative mRNA expression of osteoclast differentiation marker genes including TRAP, calcitonin receptor, V-ATPase d2, and cathepsin K was evaluated by qRT-PCR. *P<0.05 and **P<0.01 versus the pBABE group.

### Overexpression of miRNA-340 inhibited the protein level of MITF

Given that MITF functions as crucial transcription factor involved in osteoclast differentiation, many miRNAs targeting MITF were sought. By using a bioinformatics tool TargetScan (ver. 7.1, http://www.targetscan.org), we found that there are miR-340 binding sites in MITF 3′UTR. The seed region of has-miR-340 was very complementary to the position 523–529 of MITF 3′UTR. To determine the specific regulationary role of miR-340 in MITF, HEK293T cells were cultured, and cotransfected with wt or mutant MITF 3′UTR luciferase reporter plasmids, together with control mimics or miR-340 mimics. After incubation for 24 h, HEK293T cells were subjected into luciferase reporter assay. Data revealed that overexpression of miR-340 repressed the luciferase activity of wt MITF 3′UTR reporter while fails to exert obvious negative effect on mutant MITF 3′UTR reporter where the miR-340 binding site was mutated (Figure 3A). These findings suggested that MITF was a direct target of miR-340. Moreover, once the binding site present on MITF 3′UTR is mutated, the interactions between miR-340 and MITF are abolished. To further verify the negative regulation of miR-340 on MITF, BMMs were transfected with pBABE-340 vector to overexpress miR-340 and then differentiated into osteoclasts in osteoclastogenesis condition for 24 h. As shown in Figure 3(B), RT-PCR analysis showed that the relative mRNA level of MITF in BMMs transfected with pBABE-340 vector was down-regulated compared to that in BMMs transfected with the empty pBABE vector. Moreover, Western blot analysis showed that the protein expression level of MITF in BMMs transfected with pBABE-340 vector was lower than that in BMMs transfected with empty pBABE vector. Taken together, our results suggested that overexpression of miRNA-340 inhibited both the mRNA and protein expression level of MITF.

**Figure 3:** Overexpression of miR-340 inhibited the expression level of MITF (**A**) MITF was a direct target of miR-340. Alignment between the predicted has-miR-340 target sites of MITF 3′UTR and has-miR-340 was shown. HEK293T cells were subjected to luciferase reporter assay after cotransfection with wt or mutant MITF 3′UTR luciferase reporter plasmids, plus control mimics or miR-340 mimics for 24 h. (**B**) BMMs were differentiated into osteoclasts in the presence of M-CSF and RANKL for 24 h. The relative mRNA level and the protein expression level of MITF in BMMs transfected with the pBABE empty vector (control) or pBABE-340 vector was analyzed by qRT-PCR and Western blot respectively. β-actin served as the loading control in Western blot. *P<0.05 and **P<0.01 versus the pBABE group.

### Silencing MITF inhibited TRAP, calcitonin receptor, V-ATPase d2, and cathepsin K

To determine the effect of MITF on osteoclast differentiation, BMMs were transfected with negative control siRNA (control), or si-MITF. Results of qRT-PCR and Western blot revealed that both the relative mRNA and protein expression levels of MITF in BMMs were significantly decreased by siRNA-mediated inhibition of MITF expression (Figure 4A and B). In addition, qRT-PCR was performed to analyze the relative expression levels of osteoclast differentiation marker genes including TRAP, calcitonin receptor, V-ATPase d2, and cathepsin K in BMMs transfected with negative control siRNA (control) or si-MITF. Data revealed that the relative TRAP expression in BMMs transfected with si-MITF was lower than that in BMMs transfected with control siRNA, suggesting that MITF knockdown inhibited the expression of TRAP. Similar results were observed in calcitonin receptor, V-ATPase d2, and cathepsin K groups (Figure 4C). Taken together, our results indicated that silencing MITF inhibited osteoclast differentiation.

**Figure 4:** Silencing MITF inhibited TRAP, calcitonin receptor, V-ATPase d2 and cathepsin K. BMMs were differentiated into osteoclasts in the stimulation of M-CSF and RANKL (**A**) The relative mRNA level of MITF in BMMs transfected with negative control siRNA (control) or si-MITF was detected by qRT-PCR. (**B**) The protein expression level of MITF in BMMs transfected with negative control siRNA (control) or si-MITF was measured by Western blot. (**C**) The relative mRNA levels of osteoclast differentiation marker genes including TRAP, calcitonin receptor, V-ATPase d2, and cathepsin K in BMMs transfected with negative control siRNA (control) or si-MITF were examined by qRT-PCR. **P<0.01 versus the control group.

## Discussion

Accumulating evidences have discovered that osteoclast differentiation is regulated by many cytokines and transcription factors, such as M-CSF, RANKL, Src, Myc, nuclear factor (NF)-κB, NFATc1, and MITF [22]. M-CSF has been reported to be essential for osteoclast differentiation via binding to its receptor c-Fms [1,23,24]. RANKL plays prominent roles in regulating osteoclast formation on mononuclear precursors by interacting with its receptor RANK [25]. Until present, osteoclasts differentiation can be achieved with macrophages in the stimulation of M-CSF and RANKL [1,2,26], which was consistent with our findings that BMMs were differentiated into more TRAP-positive osteoclasts in the stimulation of M-CSF and RANKL compared with control BMMs, indicating the role of M-CSF and RANKL to promote osteoclastogenesis.

A large number of miRNAs play critical roles in modulating various biological processes of osteoclast differentiation and function [6]. Generally, miRNAs that decreased in expression level during osteoclast differentiation or formation tend to inhibit osteoclastogenesis, and vice versa. For instance, miR-31 was elevated during RANKL-induced osteoclastogenesis and inhibition of miR-31 impaired the osteoclast formation under RANKL induction [27]. While miR-7b was down-regulated during osteoclastogenesis in RAW264.7 cells stimulated by M-CSF and RANKL, and overexpression of miR-7b decreased TRAP-positive MNCs in number, inhibition of miR-7b promoted osteoclastogenesis [28]. Besides, Qu et al. [29] manifested that miR-218-5p acted as a negative regulator of osteoclastogenesis by targeting the p38MAPK-c-Fos-NFATc1 pathway. Chen et al. [30] also presented that miR-503 inhibited osteoclast differentiation by suppressing RANK, which was a target of miR-503. However, the association between the expression profile of miRNAs and its function in osteoclastogenesis is complicated. For example, miR-26a was up-regulated in BMMs but inhibited osteoclast formation, the opposite effect exerted by those elevated miRNAs [31]. Despite increasing researches for miRNAs in regulating bone remodeling, the precise role of miR-340 in osteoclastogenesis remains further investigation. Ma et al. [13] has reported that miR-340 could regulate RAS/RAF/mitogen-activated protein kinase (MAPK) signaling, the activation of which is crucial in osteoclastogenesis, thereby is likely to exhibit potential roles in osteoclasts [32]. Our present study demonstrated that miR-340 can be significantly decreased during osteoclast differentiation under the stimulation of M-CSF and RANKL. In addition, the relative mRNA expression level of TRAP, calcitonin receptor, V-ATPase d2, and cathepsin K was decreased in BMMs in response to overexpression of miR-340, which was consistent with the impairment of TRAP staining activity in BMMs, further verified the inhibitory effect exerted by miR-340 on osteoclast differentiation.

MiRNAs have been reported to mediate a negative regulation in gene expression after binding to 3′UTR of a target mRNA by regulating transcript localization, polyadenylation, and translation [6,7,33,34], which supported our findings that miR-340 exerted an inhibitory effect on the expression of MITF by binding to 3′UTR of MITF. MITF was established by Luchin et al. [15] for the first time to be implicated in osteoclast differentiation. MITF induces hematopoietic stem cells to differentiate into osteoclast precursors and is a pivotal transcription factor involved in the late stages of osteoclastogenesis [35]. Besides, MITF was identified to promote macrophage survival and MITFmi/mi mice exhibited severe osteopetrosis [36]. Furthermore, Mann et al. [37] stated that miR-155 suppressed the expression of MITF and thus inhibited RANKL-induced osteoclast differentiation. We herein found that MITF knockdown inhibited the expression of TRAP, calcitonin receptor, V-ATPase d2, and cathepsin K, suggesting that silencing MITF inhibited osteoclast differentiation. Taken together, we can conclude that overexpression of miR-340 inhibited osteoclast differentiation, which was likely to be mediated by repression of MITF expression.

In summary, our study showed that miR-340 inhibits osteoclast differentiation by suppressing the expression of MITF. Our findings suggest the association between miR-340 and MITF and the critical roles of them during osteoclast differentiation, which provides promising therapeutic targets for further treatment of osteoclast-related diseases.

## Abbreviations

BMM: bone marrow-derived macrophage
M-CSF: macrophage-colony stimulating factor
α-MEM: α-minimum essential medium
MITF: microphthalmia-associated transcription factor
MNC: multinucleated cell
NF: nulear factor
RANKL: receptor activator of nuclear factor-κB ligand
TRAP: tartrate-resistant acid phosphatase
wt: wild-type
